This article has been retracted.

# Elucidation of Genotypic Variability, Character Association, and Genetic Diversity for Stem Anatomy of Twelve Tossa Jute (*Corchorus olitorius* L.) Genotypes

**DOI:** 10.1155/2020/9424725

**Published:** 2020-07-23

**Authors:** Md. Mia Mukul

**Affiliations:** Scientific Officer, Breeding Division, Bangladesh Jute Research Institute (BJRI), Ministry of Agriculture, Manik Mia Avenue, Dhaka, Bangladesh

## Abstract

**Background and Aims:**

Anatomy of twelve tossa jute genotypes were performed for the variability, heritability, and genetic advance based on yield attributing six anatomical traits.

**Materials and Methods:**

The experiments were carried out in field and laboratory including 12 tossa jute genotypes followed by RCB design in JAES, Manikganj, and Bangladesh Jute Research Institute, Dhaka, Bangladesh, during 2019-2020. *Hypothesis*. The tested genotypes were expected to perform better than controls in respect of anatomical characters contributing to fiber yield in tossa jute plants.

**Results:**

Five genotypes, i.e., Acc. 1318, Acc. 1306, JRO S_1_, O-412-9-4, and O-0512-6-2 providing good results for the total fiber bundle area, trapezoid number, bark diameter, area of trapezoid, and bark thickness per transverse section in the anatomy of jute plants depicting the more variability (*P* > 0.01) as well as the possibility of tossa jute varietal development. These morphological and anatomical traits showing highly significant association (^∗∗^) with one another and coupled with high genetic and phenotypic variance components; high heritability; high and moderate genetic advance and higher divergence in clustering (*D*^2^), and PCA would be used as criteria for selection and improvement for fiber yield of tossa jute.

**Conclusions:**

The high variation and divergence for anatomical characters may be considered an effective selection method of genotypes for higher fiber yield comparing with controls. The genotypes, i.e., Acc. 1318, Acc. 1306, JRO (segregate), O-412-9-4, and O-0512-6-2 with good anatomical traits related to fiber yield could be used as parents in breeding program as well as direct variety development.

## 1. Introduction

Jute is the second most important fibrous plant after cotton throughout the world [1]. It is a natural fiber producing crop bearing chromosome number 2n = 2x = 14 belonging the genus *Corchorus* and family *Tiliaceae.* Jute fiber is a secondary phloem fiber or bast fiber obtained from the bark of the stem. The genus *Corchorus* is composed of approximately 100 species [2, 3]. Among these, two species, namely, white jute (*Corchorus capsularis* L.) and tossa jute (*Corchorus olitorius* L.), are commercially cultivated for natural fiber in areas distributed throughout the tropical and subtropical regions of the world, particularly in Asia, Africa, and Latin America [4, 5]. The *C. capsularis* is originated from Indian subcontinent and *C. olitorius* from Africa, and these are geographically distributed with wide genetic diversity [5]. The jute phloem fiber is a common source of commercial fiber, and phloem fibers are also produced from several plant species, including *C. capsularis* and *C. olitorius* (jute), *Linus usitatissimum* (flax), *Boehmeria nivea* (ramie), and others [6]. The phloem fibers are sclerenchyma cells with copious secondary wall thickening in the dicotyledonous jute plants [7]. This fiber is a completely biodegradable, recyclable, and eco-friendly lignocellulose fiber [5, 8]. Jute is a “Golden Fiber” of Bangladesh contributing about 4% GDP to the national economy and earns about 5% of the foreign exchange as well. Jute allows the selection of varieties with finer and high-quality fiber which gained considerable attention over the years in China, Bangladesh, and India [9, 10]. Jute fiber is mostly used for making gunny bags and packaging materials for agricultural and industrial products. The cultivated species of jute are globally important for fiber yield, and their wild species are potential source for abiotic and biotic stress tolerant genes as well as important genetic resources [11]. Genetic improvement of the cultivars of jute is needed to broaden the genetic base of new varieties. The two species indeed are distantly related, and their maternal origins are different. On the contrary, genetic variability present at the intraspecific level is low [12]. A severe competition between jute and synthetic fibers is going on in respect of fineness, strength, and price. The future of jute fiber is very greatly depending on its quality. Jute will never be able to win this competition unless its quality is greatly improved and ensured the grade-wise price for the users. The exploitation of existing diversity of each individual accession by using anatomical traits is an initial step towards crop improvement within short time. Nwangburuka and Denton [13] reported significant differences among fifteen tossa jute genotypes in terms of morphological traits, i.e., bark diameter, bark thickness, number of trapezoid, area of trapezoid, fiber bundle area, and number of bundle layer in a trapezoid. The breeders gather deep knowledge on the genetic diversity and variability, genetic architecture for fiber yield, and yield-related anatomical traits of jute germplasm for varietal improvement of jute [14]. To study the anatomical features of jute plant, destructive sampling is required to be done prior to seed production [15]. The plants are sometimes selected on the basis of some morphological traits which is actually unable to give any accurate information on fiber quality. So, the breeders need to do anatomical studies of jute plants for accurate information on fiber improvements [16]. The measurement of fiber qualities from textile properties after maturing of the plants, harvesting, retting, and washing and drying of fiber is a time and space-consuming tedious process. The alternative way to predict the fiber quality and yield capacity from anatomical study of plant stem was reported by Maiti [17], and it was observed that the yield as well as the fineness of fiber is directly correlated with (i) the area of the transverse section of jute stem and fiber bundle and (ii) the number of fiber bundle in the transverse section of jute stem and fiber cells per bundle. Correlations between jute fiber quality and other yield attributing anatomical characters are helpful to improve desired characters as well as to select good germplasm for breeding purpose [18, 19]. Multivariate methods such as cluster analysis and principal component analysis (PCA) have proven to be useful for characterizing, evaluating, and classifying germplasm for diversity when a large number of accessions or genotypes to be assessed for several characteristics of anatomical importance [20]. Therefore, twelve tossa jute genotypes were anatomically studied to estimate the variabilities among them; to estimate correlations among these stem anatomical traits; and to identify the genotype(s) with higher genetic diversity for use in efficient breeding programs and varietal development in the future.

## 2. Materials and Methods

### 2.1. Location of the Experiment and Plant Materials

The experiment was conducted as partly in the field of jute agricultural experiment station (JAES) at Jagir-Manikganj (23°52′56.1^″^N 90°01′53.0^″^E) District and in the laboratory of Breeding Division, Bangladesh Jute Research Institute (BJRI), Manik Mia Avenue (23°45′26^″^N, 90°22′47^″^E), Dhaka, Bangladesh, during 2019 to 2020 [21]. Twelve tossa jute genotypes were used in this experiment which are mentioned in Table 1 with all information.

### 2.2. Seed Preparation, Experimental Design, Seeding, and Plant Growing

The experimental plots were prepared by ploughing, weeding, and leveling. Fertilizers (urea, TSP, MoP, zypsum, and zinc sulphate) were applied at 100, 50, 60, 95, and 11 kg ha^−1^, respectively [22]. The seeds were treated with fungicide (Bavistin at 0.25% of seed weight) to remove seed borne pathogens and sun dried to break the dormancy [23]. Seeds of each genotype were sown in 3 m length in 5 lines with line to line 30 cm, plant to plant 8-10 cm, and genotype to genotype 80 cm distance for the experiment during summer (*Kharif*) season. Plants were grown (Figure 1) followed by agronomic practices, i.e., weeding, thinning, roguing, irrigation, fertilization, and pesticide spray.

### 2.3. Harvesting, Stem Sample Collection, Preservation, and Microscopic Study

After 120 days of sowing, 10 plants were selected randomly from the middle row of each genotype and harvested for an anatomical study. For a rapid and nondestructive anatomical study, 10 cm long stems [fiber (phloem) and stick (xylem)] were collected from the top, middle, and basal parts of each genotype. These samples were labeled and preserved in formaldehyde acetic acid (FAA) solution [formalin: acetic acid: alcohol⁃5 : 15 : 80] [24]. From these samples, transverse sections (0.15-0.20 mm thin) were made using a hand-operated Microtome machine (WSL Lab Microtome-modified Reichert-type) and the additional mucilage was removed by rinsing with clean water and then stained with 1% safranin (aqueous) solution [25] for a microscopic study. The stained sample sections were mounted with a drop of glycerin water on a glass slide with a cover slip [26]. The sections were observed under an electronic microscope, and anatomical data, i.e., bark diameter, bark thickness, height of trapezoid, width of trapezoid, area of trapezoid, number of trapezoid, fiber bundle area per section, and number of bundle layer trapezoid^−1^, were recorded carefully.

### 2.4. Statistical Parameters and Data Analyses

All the data were compiled carefully in Microsoft excel program. The analysis for variability and least significant differences (LSD) among the genotypes and significant association among all anatomical traits were estimated followed by RCBD design using statistical analysis software Statistix 10 [27] and SPSS [28]. The mean sum of square of genotype (MS_G_) and mean sum of error (MS_E_) were estimated using the analysis software. The MS_E_ was considered an error variance (*σ*_E_^2^). LSD tests were checked from a calculated and tabulated value of “*F*” at both *P* > 0.05 and *P* > 0.01 levels. Pearson's correlation coefficient among all characters in all possible combinations was estimated using the formula given by Cohen [29].

Genetic parameters like genotypic and phenotypic variances of the trait(s) were calculated using formulae (i) and (ii); and the genotypic, phenotypic, and environmental covariance components between two traits were calculated using formulae (iii)–(vii) suggested by Burton [30]; Johnson et al. [31].

(1) $$\begin{array}{c} \text{Genotypic variance }\left(\text{GV}\right)\text{: }\sigma_{\text{G}}^{2}=\frac{{\text{MS}}_{\text{G}}-{\text{MS}}_{\text{E}}}{r},\\ \text{Phenotypic variance }\left(\text{PV}\right)\text{: }\sigma_{\text{P}}^{2}=\sigma_{\text{G}}^{2}+\sigma_{\text{E}}^{2},\\ \text{Error variance}:\sigma_{\text{E}}^{2}=\frac{{\text{MS}}_{\text{E}}}{r},\\ \text{Genotypic coefficient of variation}:\text{GCV }\left(\%\right)=\frac{\sqrt{\sigma_{\text{G}}^{2}}}{\bar{X}}\times 100,\\ \text{Phenotypic coefficient of variation}:\text{PCV }\left(\%\right)=\frac{\sqrt{\sigma_{\text{P}}^{2}}}{\bar{\text{X}}}\times 100,\\ \text{Environmental coefficient of variation}:\text{ECV }\left(\%\right)=\frac{\sqrt{\sigma_{\text{E}}^{2}}}{\bar{X}}\times 100,\\ \text{Population mean of variable }\bar{X\;}\text{or }\bar{Y}=\frac{\sum_{X\text{ or }Y\text{ variable}}\left(\text{average of replicated values}\right)}{\text{Total number of observation }\left(N\right)}, \end{array}$$

where MS_G_ is the genotypic mean square value, MS_E_ is the error mean square value, *r* is the number of replication, *σ*_E_^2^ is the environmental variance (error mean square from the analysis of variance), and $\bar{X}\text{ or }\bar{Y}$ is the mean value of the trait/variable *X* or *Y* being evaluated.

#### 2.4.1. Heritability in Broad Sense, *h*_bs_^2^(%)

According to Lush [32], Johnson et al. *[*28*]*, and Burton and Devane [33], the *h*_bs_^2^(%) was estimated as follows:

(2) $$\begin{array}{c} h_{\text{bs}}^{2}=\frac{\sqrt{\sigma_{\text{G}}^{2}}}{\sqrt{\sigma_{\text{P}}^{2}}}\times 100. \end{array}$$

#### 2.4.2. Estimation of Genetic Advance (GA) and Genetic Advance in Percentage of Mean (GAM)

The expected GA for different characters under selection was estimated using formula (ix) given by Lush [32] and Johnson et al. [31].

(3) $$\begin{array}{c} \text{GA}=\frac{\sqrt{\sigma_{\text{G}}^{2}}}{\sqrt{\sigma_{\text{P}}^{2}}}\times K\times \sigma_{\text{P}}, \end{array}$$

where *K* is the selection differential (*K* = 2.06 at 5% selection intensity) and *σ*_P_ is the phenotypic standard deviation (STDEV.S) of the character.

According to Comstock and Robinson [34], genetic advance in the percentage of mean (GAM) was calculated as follows:

(4) $$\begin{array}{c} \text{GAM }\left(\%\right)=\frac{\text{GA}}{\bar{X}}\times 100, \end{array}$$

where $\bar{X}$ is the grand mean of the character.

#### 2.4.3. Correlation Coefficient (*r*_*XY*_) and Partitioning into Genotypic and Phenotypic Correlations (*r*_*G*_*XY*__ and *r*_*P*_*XY*__)

Between the variables *X* and *Y*, the variance and covariance components among the traits were computed using formulae (xi) and (xii), and Pearson's correlation coefficient among all characters in all possible combinations was estimated using formula (xiii) given by Cohen [29]. The genotypic correlation (*r*_G_*XY*__) and phenotypic correlation (*r*_P_*XY*__) for all possible combinations were estimated using these covariance components and formulae (xiv) and (xv) suggested by Karim et al. [32] and Johnson et al. [31] as follows:

(5) $$\begin{array}{c} \text{Variance }\left(\text{population}\right)\text{of variable }X\;\left(\sigma_{x}^{2}\right)=\frac{\sum_{i=1}^{N}{\left(x_{i}-\mu \right)}^{2}}{N},\\ \text{Covariance between variables }X\text{ and }Y\;\left({\text{Cov}}_{XY}\right)=\overset{N}{\underset{i=1,2,\cdots ,n}{\sum }}\frac{\left(X_{i}-\bar{X}\right)\cdot \left(Y_{i}-\bar{Y}\right)}{\text{N}-1},\\ \text{Correlation between variables }X\text{ and }Y\;\left(r_{XY}\right)=\frac{{\text{Cov}}_{XY}}{\sqrt{\sigma_{X}^{2}\times \sigma_{Y}^{2}}},\\ \text{Genotypic correlation between variables }X\text{ and }Y\;\left(r_{{\text{G}}_{XY}}\right)=\frac{{\text{Cov}}_{\text{G}}XY}{\sqrt{\sigma_{\text{G}}^{2}\;X\times \sigma_{\text{G}}^{2}\;Y}},\\ \text{Phenotypic correlation between variables }X\text{ and }Y\;\left(r_{{\text{P}}_{XY}}\right)=\frac{{\text{Cov}}_{\text{P}}XY}{\sqrt{\sigma_{\text{P}}^{2}\;X\times \sigma_{\text{P}}^{2}\;Y}}, \end{array}$$

where *N* is the number of observation in variable *X* or *Y*.

#### 2.4.4. Genetic Divergence

Genetic divergence plays a vital role in existing germplasm in the mode and source of origin. It also measures the distance for a number of traits between two populations. The genotypes were grouped based on Euclidean squared distances (*D*^2^) and Ward's method as described by Joe [36].

#### 2.4.5. *D*^2^ Values

The Mahalanobis distance (*D*^2^) values were calculated from the transformed uncorrelated means of characters [37, 38]. For each combination, the mean deviation, *Y*_*i*_^1^–*Y*_*i*_^2^ with *i* = 1, 2, ⋯, *p*, was estimated, and the *D*^2^ value was calculated as the sum of squares of these deviations, that is, *Σ*(*Y*_*i*_^1^–*Y*_*i*_^2^)^2^. The *D*^2^ values were estimated for all possible pairs of combinations between genotypes.

#### 2.4.6. Clustering

The D^2^ values of genotypes were arranged in order of relative distances from each other [37], while the method suggested by Singh and Chaudhary (1985) was used for cluster formation.

#### 2.4.7. Average Intra- and Intercluster Distances

Average intra- and intercluster distances were calculated by the following formula ([38]):

(6) $$\begin{array}{c} \text{Average intracluster}:D^{2}=\frac{\sum D^{2}}{n},\\ \text{Average intercluster}:D^{2}=\frac{\sum D^{2}\;ij}{ni\times nj}. \end{array}$$

#### 2.4.8. Clustering and Principal Component Analysis (PCA)

Principal component analysis (PCA) is a technique for reducing the dimensionality of large datasets, increasing interpretability but at the same time minimizing information loss [39]. It does so by creating new uncorrelated variables that successively maximize variance. Finding new variables with the maximum variance, the principal components, reduces to solve an eigenvalue problem, and the new variables are defined by the dataset at hand, hence making PCA an adaptive data analysis technique [39]. *D*^2^ statistics, cluster mean analysis, and two-dimensional principal component analysis were carried out by using statistical software package Minitab19 [40].

## 3. Results and Discussion

### 3.1. Anatomy of Tossa Jute Plant

The jute fibers obtained from the stem (commercially known as bast fibers) lie embedded in the softer tissue of the bark [41]. The jute fibers lie within the stem of the plant just beneath the bark and surrounded by the soft tissue [42]. This type of bast fiber is known as a phloem fiber which is derived from cambial meristematic activity which cuts fiber initials that grow longitudinally along the axis within the bark. Each of these cells, pointed at both ends with a lumen at the center, is called an ultimate fiber cell (Figures 2, 3(a) and 3(b)).

#### 3.1.1. Analyses of Variance (ANOVA)

The analyses of variance revealed significant differences for anatomical characters along with plant height, stem base diameter, and yield content indicating the presence of variability among all tossa jute genotypes (Table 2). The mean values of different anatomical characters were estimated (Table 3), and the patterns of fiber development in 12 tossa jute genotypes were studied (Figures 4(a)-4(l)). Maity et al. [11] firstly proposed the possibility of prediction of fiber quality and yield capacity from the anatomy of jute plant.

#### 3.1.2. Bark Diameter

In the anatomy of jute plants (Figures 4(a)-4(l)), the highest bark diameters were recorded in Acc. 1318 at the plant base, middle, and full plant (7.56, 14.78, and 13.35 mm, resp.) and 7.89 mm at middle of stem in O-043-7-9. Considering full plant, the good results for bark diameter were found in Acc. 1318 (13.35 mm), JRO (segregate) (11.59 mm), and Acc. 1306 (11.30) than control varieties (Table 3; Figures 4(b), 4(i), and 4(a)). These materials would be used as parent material in hybridization program. Jute genotypes with higher bark diameter contribute to fiber (phloem) and stick (xylem) yield [43].

#### 3.1.3. Bark Thickness

The space between the upper surface of cambium cell and the epidermis of phloem tissue is known as the bark thickness of jute plant. Phloem fibers or bast fibers are made up of sclerenchymatous cells (Figure 3) which are generally absent in primary phloem but are found in the secondary phloem [44]. The highest bark thickness at the base, middle, and top of the plants was found in JRO (segregate) (4.55 mm), Acc. 1318 (3.91 mm), and O-043-7-9 (2.37) (Figures 4(i), 4(b), and 4(f), resp.). In the full plant, the highest bark thickness was recorded in Acc. 1318 (3.42 mm) followed by JRO (segregate) (3.24 mm) and Acc. 1306 (3.17 mm) compared to controls (Table 3; Figures 4(b), 4(i), and 4(a)). Bark thickness is an important criterion for the phenotypic selection of breeding materials in jute plant breeding approaches [43].

#### 3.1.4. Area of a Trapezoid

The highest area of a trapezoid was found in Acc. 1318 (Figure 4(b)) at base (0.53sqmm), top (0.51sqmm), middle (0.27sqmm), and overall full plant (0.43 sqmm) followed by Acc. 1306 (0.41sqmm) than the control varieties (Table 3). The jute genotypes with maximum area of a trapezoid contribute to higher fiber yield, and these genotypes would be used as parent(s) for hybridization purposes [45].

#### 3.1.5. Average Number of Trapezoid

The average number of trapezoid was found to be higher in the transverse section of BJRI tossa pat-5 at base (78.33); in Acc. 1318 at middle (66.67) and full plant (60.56); and in top of O-049-1-3 (51.67). Considering the full plant, the Acc. 1318, O-049-1-3, and O-0512-6-2 gave the good results for trapezoid number (60.56, 59.33, and 57.56; Figures 4(b), 4(g), and 4(c), resp.) in the transverse section of jute plant (Table 3). Jute genotype(s) with higher plant height and base diameter gave maximum number of trapezoid per transverse section. The maximum number of trapezoid gives more area of fiber bundle. These results were corroborated by Oram et al. [46]. So, the Acc. 1318 will be considered a good genotype in respect of trapezoid number as well as fiber bundle area.

#### 3.1.6. Fiber Bundle Area

It was found that Acc. 1318 gave higher fiber bundle area in transverse section at the middle (33.98 mm) and top (11.33 mm) of jute stem, also considering the full plant (27.88 mm). BJRI tossa pat-5 showed the highest fiber bundle area (39.16 mm) at base of the stem. In respect of full plant, the fiber bundle area recorded in Acc. 1318 (27.88 mm) and Acc. 1306 (22.95 mm) which were higher than all controls (Table 3; Figures 4(b) and 4(a)). The bark diameter, bark thickness, number of trapezoid, and area of trapezoid contributing to total fiber bundle area in jute plant would be the criteria for phenotypic selection for fiber yield [16, 47].

#### 3.1.7. Fiber Bundle Layer in Trapezoid

Maximum fiber bundle layer trapezoid^−1^ was found in transverse section at the base of BJRI tossa pat-5 (13.22), at the middle of Acc. 1318 (9.44), and at the top of O-043-7-9 (5.22). In the full plant, the highest fiber bundle layer trapezoid^−1^ was found in JRO (segregate) followed by Acc. 1318 (8.56) and O-049-1-3 (8.19) (Table 3). The number of fiber bundle layer in trapezoid contributes to fiber bundle area as well as the fiber yield in jute plant [48].

#### 3.1.8. Plant Height Performance

Among all genotypes, the genotype Acc. 1306 showed the highest plant height (3.22 m), and O-049-1-3, Acc. 1306, O-0512-6-2, BJRI tossa pat-5 showed almost similar results for plant height (Table 4). The genotypes with higher plant height compared to controls would be used as breeding materials to develop a new variety which was also corroborated by Zhang et al. [49].

#### 3.1.9. Plant Stem Base Diameter Performance

The plant with a higher base diameter is important for fiber crops. The fiber is mainly produced from the basal and middle portion of the plant. In this investigation, Acc. 1318 gave a maximum base diameter (16.63 mm) with higher fiber content followed by O-049-1-3, O-0512-6-2, JRO-524, O-0411-10-4, and O-0419-3-1 compared to controls BJRI tossa pat-5 and BJRI tossa pat-8 (Table 4). The highest diameter with more fiber (phloem) content at the base of the tossa jute plant contributes to fiber yield content and could be used for varietal development; it was agreed with Zhang et al. [49].

#### 3.1.10. Fiber Yield Performance

A higher fiber yield is the main objective of jute plant. The genotype Acc. 1318 gave higher fiber yield (3.55 t ha^−1^) followed by Acc. 1306, O-0512-6-2, JRO-524, BJRI tossa pat-5, JRO (segregate), and O-0411-10-4. For fiber content, Acc. 1318, Acc. 1306, and O-0512-6-2 performed well than the controls (Table 4). These genotypes would be further cultivated for the next generation to develop high yielding new varieties. The jute breeding materials as well as the hybridized offspring(s) providing higher fiber content are generally considered for developing high yielding varieties of jute crop [50]. Jute sticks are useful materials which are now used in various aspects to produce charcoal, desk board of valuable cars, and ink [51]. From this study, the genotypes (Acc. 1318, Acc. 1306, O-0512-6-2, O-0411-10-4, and O-049-1-3) giving higher stem height, base diameter, and fiber content showed higher stick yield per plant compared to controls (Table 4).

### 3.2. Correlation Coefficients for Anatomical Characters and Partitioning into Genotypic and Phenotypic Levels

The anatomical characters of 12 jute plants showed highly significant and positive correlations (2 tailed) with one another, where the average number of trapezoid per transverse section showed significant relation with other characters at general level (Table 5) as well as genotypic and phenotypic levels (Table 6) and nonsignificantly associated with area of trapezoid at phenotypic level (Table 6). The bark thickness, area of a trapezoid, number of trapezoid, and number of fiber bundle layer in trapezoid contribute to total fiber bundle area in jute stem as well as fiber and stick yield in jute plants. These anatomical features would be the selection criteria to the jute breeders for jute crop improvement in Bangladesh [52].

### 3.3. Distribution of Fiber Cells in Cross Section of Different 12 Tossa Jute Genotypes at Stem Base

### 3.4. Heritability, Genetic Variances, Covariances, and Advances for Anatomical Characters

The analyses for genetic parameters of six anatomical characters of jute plant (Table 7) revealed that the genotypic and phenotypic variances (*σ*_G_^2^, *σ*_P_^2^) were ranged from 0.003 to 19.587 and from 0.004 to 21.975 for the area of a trapezoid and the average number of trapezoid T.section^−1^. The genotypic, phenotypic, and environmental covariances (GCV, PCV, and ECV) were ranged from 2.332 to 19.985%, from 2.455 to 22.374%, and from 0.942 to 12.323% for bark thickness and total fiber bundle in the jute plants. The GCV values were higher than the PCV values for all anatomical characters. The ECV values were found very lowest for all characters indicating the lower effects of environmental factors on jute plant growth. All the traits showed high heritability (>80%) where the highest value (99.449) was recorded in the bark diameter and lowest (86.874) in the area of a trapezoid. The highest genetic advance was found in the average number of trapezoid per T.section (8.866) followed by the total fiber bundle area per T.section (7.252) indicating the possibility of increasing these traits from 18.58 to 25.832 sqmm total fiber bundle area and from 54.08 to 62.946 number of trapezoid section^−1^ contributing to fiber yield improvement in jute plants.

The genetic advance in the percent of mean ranged from 4.684% to 39.032% for bark diameter and total fiber bundle area section^−1^. Johnson et al. [31] categorized the value of GAM as low (<10%), moderate (10–20%), and high (>20%). Accordingly, the GAM values for the total fiber bundle area section^−1^, area of a trapezoid, and bark diameter were categorized as high; for the average number of trapezoid section^−1^ and bundle layer trapezoid^−1^ were categorized as medium; and for the bark thickness was low. The characters having high to medium GAM values indicate the greater possibility of improvement for these characters as well as fiber yield of the jute plants. High *h*_bs_^2^ along with the GAM is usually more helpful in predicting gain under selection than heritability alone. The total fiber bundle area in transverse section coupled with higher GV, PV, GCV, PCV, *h*_bs_^2^, GA, and GAM would be the principal selection criteria for improving fiber yield in jute plants which was agreed with the findings of Islam et al. [53].

### 3.5. Hierarchical Cluster Analysis

Cluster analysis using all anatomical traits grouped all genotypes into four major clusters at the genetic distance of 77.50 (Figure 5) and indicates that twelve tossa jute genotypes exhibited notable genetic divergence in terms of anatomical traits [54]. The dendrogram tends to group some of the genotypes with similar anatomical traits into the same cluster. It was also found that, among the four clusters, cluster III was the largest and consisted of 7 genotypes (58.33%) including 5 breeding lines and two controls, i.e., BJRI tossa pat-8 and JRO-524, and the second largest cluster I consisted of 3 genotypes (25.00%) including two breeding lines and one control BJRI tossa pat-5 (Table 8). Each of the other two clusters (II and IV) contained single genotype (8.33%) where cluster II contained the superior accession (Acc. 1318) and cluster IV contained the good breeding line (O-0412-9-4) with higher genetic distances from other clusters (Table 8, Figures 5 and 6).

Cluster analysis using a dendrogram and PCA following two-dimensional method played a complementary role to each other with little inconsistencies in respect of the number of genotypes in cluster formation [54]. To obtain greater heterosis, genotype(s) having distant cluster(s) could be used as parents in hybridization program or could be used to develop new high yielding variety. Dendrogram and two-dimensional PCA graph clearly indicated that the accession G_2_ = Acc.1318 and the breeding line G_4_ = O-0412-9-4 made their individual clusters (clusters II and IV) and were far away from the other two clusters. Therefore, the genotypes from clusters II and IV could be used for varietal the development program of tossa jute in Bangladesh. Similar findings were reported in soybean plant by Malek et al. [54].

### 3.6. Cluster Mean Analysis

This character is more important as it is closely associated with fiber fineness. The mean values of six different anatomical traits for four clusters among twelve tossa jute genotypes (Table 9) showed that cluster II had the highest average means for all anatomical traits. On the contrary, cluster III revealed the lowest mean values for bark diameter and bark thickness, and cluster IV showed lower values for area of trapezoid, number of trapezoid, fiber bundle area, and fiber bundle layer in the transverse section of jute plants. Based on the mean values, clusters I and II showed good results for all traits, and the average number of trapezoid per section showed good records in cluster III, also (Table 9). The mean values for total bundle area per section were high in cluster II (8.556 sqmm), medium in cluster II (8.346 sqmm), and lower in cluster V (7.097 sqmm). Similar kinds of results were reported by Ghosh et al. *[*51*]* while working on jute crop.

### 3.7. Cluster Distance (*D*^2^) Analysis

Intra- and intercluster distances for similarity and dissimilarity among twelve tossa jute genotypes were estimated using Ward's method (Figure 6). The higher intercluster distance (7.01) was recorded between cluster II and cluster IV, while the minimum distance (2.81) was found between cluster III and cluster IV and medium distance (4.12) between cluster I and IV. The intracluster distances were 3.53, 0.00, 10.14, and 0.00 for clusters I, II, III and IV, respectively (Figure 6). The intracluster distances in both cluster II and cluster IV were 0.00 due to the single genotype in each cluster. The higher intercluster distances indicate the presence of high genetic divergence between the clusters; similar results were reported in tossa jute while estimating genetic diversity [56]. Selecting tossa jute genotypes from high inter cluster distances with high mean values for fiber yielding characters will help in developing high heterotypic hybrids and are also useful in selecting better recombinants in the segregating generations for higher fiber yield. In the present study, the highest intracluster distances were recorded in cluster III (10.138), indicating high variation among the genotypes in the cluster and lowest in cluster I (3.530) indicating less variation among the genotypes in this cluster. The average intercluster distances were higher than the average intracluster distances, which indicates the presence of wide genetic diversity among the genotypes of different clusters than those of the same cluster [57].

### 3.8. Principal Component Analysis (PCA)

A two-dimensional principal component analysis (PCA) was performed using all the morphological traits. The cluster analysis was mostly confirmed by the PCA (Figures 7 and 8). The eigenvalues, variabilities, cumulative variabilities, and eigenvectors of the variables among the components in PCA were shown in scree plot analysis (Table 10, Figure 7). The variabilities were increased with increasing the eigenvalues, but the variation in cumulative variabilities is vice versa (Figure 7). The first two principal components accounting for 85.80% of the total variation among the tossa jute genotypes were assessed for six anatomical characters. The first principal components explained variance about 71.00%, the second 14.80%, the third 6.80%, the fourth 5.70%, the fifth 1.40%, and the sixth 0.30% of the total variance (Figure 7); similar results were reported by Nwangburuka and Denton [13] and Ghosh et al. *[*54*]* in jute crop. The tested lines were categorized into six groups in the two-dimensional plot of PCA (Figure 8). The genotype G_2_ = Acc. 1318 and the line G_4_ = O-0412-9-4 formed their individual group (groups III and IV, resp.) in PCA; and individual clusters (clusters II and IV, resp.) in cluster analysis. The segregate G_9_ = JRO (segregate) and the accession G_1_ = Acc. 1306 of cluster I formed group I in PCA. The control variety G_10_ = BJRI tossa pat-5 of cluster I formed individual group II. The five breeding lines, i.e., G_3_ = O-0512-6-2, G_5_ = O-0411-10-4, G_6_ = O-043-7-9, G_8_ = O-0419-3-1, and G_7_ = O-049-1-3, and two control varieties, i.e., G_11_ = BJRI tossa pat-8 and G_12_ = JRO-524 under cluster III formed group IV in PCA. Characters are having high vector values closer to one within the given principal component and influence the cluster more than the variables having low values closer to zero [13]. In the 1^st^ principal component, all the traits recorded positive values, where bark diameter, bark thickness, area of trapezoid, and bundle layer in trapezoid showed higher vector values, and the other characters the number of bundle layer and fiber bundle area showed the lowest vector values. In PCII, the number of bundle layer and fiber bundle area showed positive values, and other characters recorded negative values (Table 10). Similar kinds of results were reported by Nwangburuka and Denton [13].

## 4. Conclusion

The variabilities existing among the tested genotypes for the studied anatomical traits indicate the high possibility for jute crop improvement through breeding techniques. The jute genotypes, i.e., Acc. 1318, Acc. 1306, O-0512-6-2, JRO (segregate), and O-0412-9-4, provided good results for total fiber bundle area in the transverse section, average number of trapezoid in the T.section, bark diameter and bark thickness in an anatomical study, and higher divergence in cluster and PCA depicting the variability as well as possibility of tossa jute improvement. The anatomical characters, i.e., bark diameter, bark thickness, area of trapezoid, average number of trapezoid, and fiber bundle area per section, showing significant association with one another and coupled with high genetic and phenotypic variance-covariance components, high heritability, high and moderate genetic advance, and genetic advance in the percent of mean would be used for the selection of jute genotypes as well as jute crop improvement for fiber yield. The anatomical characters may be considered an easy and effective method for screening genotypes within a short time than the morphological study. In general, the study revealed that direct selection scheme would be more promising and encouraging than indirect selection for improving yield. This could be the nature of wild accessions or advanced breeding lines because of their better adaptive traits to variable environmental conditions which have important implications for sustainable jute cultivation.

## Figures and Tables

**Figure 1:** Growing of experimental tossa jute plants.

**Figure 2:** (a) Anatomy of the jute stem [42] and (b) pattern of fiber cell distribution in cross section of jute plant [15]. FB: fiber bundle; Ep: epidermis; CT: cortex; A: total bark diameter; B: difference between fiber wedge tip; C: average length of fiber bundle; D: average width of fiber bundle at base; F: average width of fiber bundle at top; G: average width of fiber bundle at middle.

**Figure 3:** (a, b) Zoomed in view of schlerenchymatous fiber cells (phloem fiber) of tossa jute plant.

**Figure 4:** (a–l) Anatomical features of selected 12 tossa jute genotypes at stem base.

**Figure 5:** Dendrogram showing the relationships among 12 tossa jute genotypes for six anatomical characters contributing to fiber yield.

**Figure 6:** Cluster diagram showing the average intra- and intercluster distances ($D=\sqrt{D^{2}}$ values) of 12 tossa jute genotypes for six anatomical characters contributing to fiber yield.

**Figure 7:** Scree plot in PCA analysis for eigenvalues, variability (%), and cumulative variability (%).

**Figure 8:** Two-dimensional plot of PCA showing relationships among 12 tossa jute genotypes using six anatomical characters attributing to fiber.

**Table 1:** List of plant materials with their identifying characters, plant type, and source of collection.

SL	Genotype	Identifying characters	Plant type	Source
1	G_1_ = Acc.1306	Full green plant, ovate lanceolate leaf	Accession	Gene Bank, BJRI
2	G_2_ = Acc.1318	Full green plant, ovate lanceolate leaf		
3	G_3_ = O-0512-6-2	Full green plant, lanceolate leaf	True breeding lines	Breeding division, BJRI
4	G_4_ = O-0412-9-4	Stem & leaf stipule red, ovate lanceolate leaf		
5	G_5_ = O-0411-10-4	Stem & leaf stipule red, ovate lanceolate leaf		
6	G_6_ = O-043-7-9	Stem & leaf stipule red, narrow lanceolate leaf		
7	G_7_ = O-049-1-3	Stem & leaf stipule red, lanceolate leaf		
8	G_8_ = O-0419-3-1	Stem, leaf stipule & petiole red; ovate lanceolate leaf		
9	G_9_ = JRO (segregate)	Stem, leaf stipule & petiole reddish; ovate lanceolate leaf	Segregate	
10	G_10_ = BJRI tossa pat-5 (O-795)	Stem, leaf stipule & petiole red; ovate leaf	Controls (released variety)	Gene Bank, BJRI
11	G_11_ = BJRI tossa pat-8 (Robi-1)	Stem, leaf stipule & petiole reddish, lanceolate leaf with glossy surface		
12	G_12_ = JRO-524 (Navin)	Full green plant, lanceolate leaf		

**(a):** 

Traits	Plant	Genotype (d.f. = 11)	Replication (d.f. = 2)	Error (d.f. = 22)	Traits	Plant	Genotype (d.f. = 11)	Replication (d.f. = 2)	Error (d.f. = 22)
Bark diameter (mm)	Base	10.70^∗∗^	0.70	0.99	Number of trapezoid section^−1^	Base	135.85^∗∗^	67.86	27.92
	Middle	6.03^∗∗^	1.02	0.35		Middle	61.84^∗∗^	18.11	17.41
	Top	1.80^∗∗^	0.10	0.18		Top	509.87^∗∗^	11.11	14.51
	Overall	3.80^∗∗^	0.09	0.02		Overall	62.34^∗∗^	6.30	3.58
Bark thickness (mm)	Base	0.57^∗∗^	0.12	0.05	Total bundle area (sqmm) section^−1^	Base	161.95^∗^	94.44	51.57
	Middle	0.49^∗∗^	0.01	0.02		Middle	97.50^∗∗^	9.19	15.85
	Top	0.19^∗∗^	0.002	0.01		Top	14.40^∗∗^	2.38	2.00
	Overall	0.19^∗∗^	0.01	0.01		Overall	46.60^∗∗^	6.49	5.24
Area of a trapezoid (sqmm)	Base	0.03∗	0.01	0.008	Bundle layer trapezoid^−1^	Base	4.22^∗∗^	0.886	0.24
	Middle	0.02^∗∗^	0.001	0.004		Middle	1.95^∗∗^	0.063	0.17
	Top	0.01^∗∗^	0.004	0.001		Top	1.06^∗∗^	0.307	0.06
	Overall	0.01^∗∗^	0.001	0.001		Overall	0.97^∗∗^	0.27	0.05

**(b):** 

SV	d.f.	Plant height (m)	Plant base diameter (mm)	Dry fiber yield (g plant^−1^)	Dry fiber yield (t ha^−1^)	Jute stick yield (g plant^−1^)
Genotype	11	0.07^∗∗^	4.95^∗∗^	15.74^∗∗^	0.74^∗∗^	201.55^∗∗^
Replication	2	0.01	1.29	3.32	0.12	27.3
Error	22	0.002	0.47	0.44	0.02	4.03
Total	35	—	—	—	—	—
CV (%)		1.47	4.43	5.50	5.02	5.25

**(a):** 

Lines/variety	Bark diameter (mm) of jute stem				Bark thickness (mm) of jute plant				Area of a trapezoid (sqmm) in trans. section			
	Base	Middle	Top	Overall	Base	Middle	Top	Overall	Base	Middle	Top	Overall
Acc. 1306	14.33	12.06	7.50	11.30	4.21	3.17	2.12	3.17	0.51	0.45	0.26	0.41
Acc. 1318	17.56	14.78	7.72	13.35	4.00	3.91	2.34	3.42	0.53	0.51	0.27	0.43
O-0512-6-2	14.00	10.44	7.44	10.63	3.61	2.84	2.17	2.87	0.30	0.28	0.20	0.26
O-0412-9-4	14.07	10.47	7.52	10.69	3.64	2.85	2.19	2.89	0.31	0.31	0.21	0.28
O-0411-10-4	13.00	10.44	5.44	9.63	3.58	2.66	1.64	2.63	0.52	0.31	0.16	0.33
O-043-7-9	12.22	10.39	7.89	10.17	3.27	2.74	2.37	2.79	0.39	0.31	0.24	0.31
O-049-1-3	13.39	10.17	7.22	10.26	3.56	2.83	2.11	2.83	0.42	0.22	0.22	0.29
O-0419-3-1	11.39	9.22	6.83	9.15	3.37	2.42	2.13	2.64	0.33	0.28	0.27	0.29
JRO (segregate)	15.44	11.56	7.78	11.59	4.55	2.95	2.22	3.24	0.53	0.31	0.22	0.35
BJRI tossa pat-5	15.44	11.56	5.83	10.94	4.31	3.01	1.65	2.99	0.50	0.36	0.16	0.34
BJRI tossa pat-8	10.61	10.22	7.56	9.46	4.22	2.32	2.07	2.87	0.47	0.23	0.22	0.31
JRO-524	13.44	10.39	6.89	10.24	3.32	2.74	1.75	2.60	0.33	0.31	0.14	0.26
Range	6.95	5.56	2.45	4.2	1.28	1.59	0.73	0.82	0.23	0.29	0.13	0.17
Mean	13.74	10.98	7.14	10.62	3.80	2.87	2.06	2.91	0.43	0.32	0.21	0.32
S.E.	0.81	0.48	0.35	0.117	0.18	0.13	0.09	0.084	0.07	0.05	0.02	0.030
CV (%)	7.25	5.40	5.99	1.35	5.71	5.36	5.44	3.52	21.15	19.71	13.97	11.26
LSD (0.05)	1.67∗∗	1.00∗∗	0.72∗∗	0.243∗∗	0.37∗∗	0.26∗∗	0.19∗∗	0.17∗∗	0.15∗	0.11∗∗	0.05∗∗	0.06∗∗

**(b):** 

Lines/ variety	Average no. of trapezoid per trans. section of stem				Total fiber bundle area (sqmm) in trans. section of stem				Fiber bundle layer in trapezoid			
	Base	Middle	Top	Overall	Base	Middle	Top	Overall	Base	Middle	Top	Overall
Acc. 1306	70.67	50.67	37.33	52.89	36.19	22.91	9.76	22.95	11.11	8.67	4.00	7.93
Acc. 1318	72.33	66.67	42.67	60.56	38.33	33.98	11.33	27.88	11.67	9.44	4.56	8.56
O-0512-6-2	71.00	59.67	42.00	57.56	21.35	16.63	8.22	15.40	9.56	7.11	4.22	6.96
O-0412-9-4	69.33	59.67	0.42	43.14	21.67	16.93	7.66	15.42	9.73	7.29	4.27	7.10
O-0411-10-4	61.00	56.33	36.33	51.22	31.99	17.56	5.87	18.47	11.44	7.89	3.11	7.48
O-043-7-9	60.67	56.67	43.67	53.67	23.67	17.32	10.79	17.26	10.11	7.44	5.22	7.59
O-049-1-3	67.33	59.00	51.67	59.33	28.50	12.98	11.13	17.54	11.89	7.67	5.00	8.19
O-0419-3-1	60.67	59.67	43.33	54.56	20.06	16.70	11.32	16.03	10.22	7.11	4.67	7.33
JRO (segregate)	64.00	49.67	45.00	52.89	34.16	15.25	9.81	19.74	12.67	8.56	4.89	8.70
BJRI tossa pat-5	78.33	57.33	36.33	57.33	39.16	20.53	5.68	21.79	13.22	8.11	3.89	8.41
BJRI tossa pat-8	54.67	53.33	47.33	51.78	25.78	12.13	10.37	16.09	12.44	6.56	4.56	7.85
JRO-524	60.33	56.67	45.00	54.00	19.51	17.32	6.18	14.34	11.33	7.44	3.78	7.52
Range	23.66	17	51.25	17.42	19.65	21.85	5.65	13.54	3.66	2.88	2.11	1.74
Mean	65.86	57.11	39.26	54.08	28.36	18.35	9.01	18.58	11.28	7.77	4.35	7.80
S.E.	4.31	3.41	3.11	1.545	5.86	3.25	1.15	1.870	0.40	0.33	0.20	0.19
CV (%)	8.02	7.31	9.70	3.50	25.32	21.69	15.69	12.33	4.29	5.27	5.76	2.91

**Table 4:** Mean performance of 12 tossa jute genotypes for plant height, stem base diameter and yield content.

Variety/lines	Plant height (m)	Base diameter (mm)	Dry fiber yield (g plant^−1^)	Dry fiber yield (t ha^−1^)	Jute stick yield (g plant^−1^)
Acc. 1306	3.15^a,b,c^	15.40^b^	13.83^b^	3.45^b^	51.40^a^
Acc. 1318	3.22^a^	16.63^a^	16.93^a^	3.55^a^	52.70^a^
O-0512-6-2	3.15^b,c^	16.22^a,b^	13.50^b^	3.38^b^	40.40^b^
O-0412-9-4	2.73^h^	14.00^c^	9.20^f^	2.27^g^	35.00^c^
O-0411-10-4	2.95^f^	16.13^a,b^	12.10^c,d^	3.00^d^	40.00^b^
O-043-7-9	2.88^f,g^	15.60^a,b^	10.13^e,f^	2.50^f,g^	34.80^c^
O-049-1-3	3.18^a,b^	16.23^a,b^	11.07^d,e^	2.92^d,e^	39.40^b^
O-0419-3-1	3.10^c,d,e^	16.07^a,b^	9.63^f^	2.71^e,f^	37.00^b,c^
JRO (segregate)	3.04^e^	15.40^b^	12.23^c^	3.05^c,d^	38.20^b,c^
BJRI tossa pat-5	3.13^b,c,d^	15.13^b,c^	13.20^b,c^	3.30^b,c^	22.80^e^
BJRI tossa pat-8	2.84^g^	12.00^d^	11.50^d,e^	2.80^e,f^	29.00^d^
JRO-524	3.07^d,e^	16.20^a,b^	13.43^b^	3.35^b^	38.20^b,c^
Maximum	3.22	16.63	16.93	3.55	52.70
Mean	3.04	15.42	12.06	3.02	38.24
LSD _(0.05)_	0.07^∗∗^	1.16^∗∗^	1.12^∗∗^	0.26^∗∗^	3.40^∗∗^
CV (%)	1.47	4.43	5.50	5.02	5.25
$\bar{x}\pm \text{SE}$	3.04 ± 0.025	15.42 ± 0.39	12.06 ± 0.38	3.02 ± 0.09	38.24 ± 1.16

CV (coefficient of variation) = (√EMS/mean) × 100; LSD (0.05): least significant difference at 5% probability level; values with the same letters are statistically insignificant for the same variable.

**Table 5:** Correlation coefficients among anatomical traits considering the full plant.

Traits	BT	AT	AnTS^−1^	TBAS^−1^	BLT^−1^
BDM	0.899^∗∗^	0.711^∗∗^	0.340^∗^	0.812^∗∗^	0.593^∗∗^
BT		0.793^∗∗^	0.264^∗^	0.820^∗∗^	0.692^∗∗^
AT			0.262^∗^	0.948^∗∗^	0.665^∗∗^
AnTS^−1^				0.444^∗^	0.460^∗^
TBAS^−1^					0.714^∗∗^

**Table 6:** Partitioning of genotypic and phenotypic correlation coefficients among anatomical traits.

Characters	Corr.	BT	AT	AnTS^−1^	TBAS^−1^	BLT^−1^
BDM	*r*_*g*_	0.926^∗∗^	0.768^∗∗^	0.352^∗^	0.864^∗∗^	0.610^∗∗^
	*r*_*g*_	0.874^∗∗^	0.664^∗∗^	0.330^∗^	0.767^∗∗^	0.576^∗∗^
BT	*r*_*g*_		0.876^∗∗^	0.279^∗^	0.893^∗∗^	0.730^∗∗^
	*r*_*g*_		0.723^∗∗^	0.250^∗^	0.758^∗∗^	0.658^∗∗^
AT	*r*_*g*_			0.292^∗^	0.916^∗∗^	0.738^∗∗^
	*r*_*g*_			0.240	0.841^∗∗^	0.608^∗∗^
AnTS^−1^	*r*_*g*_				0.486^∗∗^	0.487^∗∗^
	*r*_*g*_				0.410^∗^	0.436^∗^
TBAS^−1^	*r*_*g*_					0.779^∗∗^
	*r*_*g*_					0.660^∗∗^

BDM: bark diameter (mm); BT: bark thickness (mm); AT: area of a trapezoid (sqmm); AnTS^−1^: average no. of trapezoid per T.section; TBAS^−1^: total bundle area per T.section (sqmm); BLT: no. of bundle layer trapezoid^−1^; ∗ and ∗∗ denote the correlation is significant at 0.05 and 0.01 probability levels.

**Table 7:** Variance, covariance, heritability, and genetic advances of anatomical traits studied.

Characters	GV (*σ*_G_^2^)	PV (*σ*_P_^2^)	GCV (%)	PCV (%)	ECV (%)	*h*_bs_^2^	GA	GAM (%)
BDM	1.261	1.275	10.572	10.631	1.365	99.449	2.306	21.717
BT	0.061	0.068	2.332	2.455	0.942	94.972	0.497	4.684
AT	0.003	0.004	16.137	18.576	11.267	86.874	0.099	31.092
AnTS^−1^	19.587	21.975	8.184	8.668	3.499	94.412	8.866	16.394
TBAS^−1^	13.787	17.282	19.985	22.374	12.323	89.319	7.252	39.032
BLT	0.307	0.341	7.100	7.483	2.895	94.879	1.112	14.255

GV: genotypic variance; PV: phenotypic variance; GCV, PCV, ECV: genotypic, phenotypic, and environmental coefficients of variation; *h*_bs_^2^: heritability in broad sense; GA: genetic advance; GAM: genetic advance in the percentage of mean; T.section: transverse section.

**Table 8:** Clustering of twelve tossa jute genotypes based on anatomical traits contributing to fiber yield.

Cluster	Number of genotypes	Genotype (%)	Genotypes
I	3	25.000	G_1_ = Acc. 1306, G_9_ = JRO (segregate), G_10_ = BJRI tossa pat-5
II	1	8.333	G_2_ = Acc. 1318
III	7	58.333	G_3_ = O-0512-6-2, G_5_ = O-0411-10-4, G_6_ = O-043-7-9, G_11_ = BJRI Tossa pat-8, G_8_ = O-0419-3-1, G_12_ = JRO-524, G_7_ = O-049-1-3
IV	1	8.333	G_4_ = O-0412-9-4
4 clusters	8 genotypes	100.00%	8 genotypes

**Table 9:** Mean values of four clusters for seven anatomical characters contributing to fiber yield.

Characters	Cluster I	Cluster II	Cluster III	Cluster IV	Mean
BDM (mm)	11.278	13.352	9.880	10.686	11.299
BT (mm)	3.134	3.418	2.734	2.892	3.044
AT (sqmm)	0.366	0.435	0.294	0.277	0.343
AnTS^−1^	54.370	60.556	53.797	43.140	52.966
TBAS^−1^ (sqmm)	8.346	8.556	7.457	7.097	7.864
BLT	21.494	27.880	16.265	15.421	20.265

**Table 10:** Eigenvalue, variability, cumulative variability, and eigenvectors of the variables among the components in PCA.

	Components					
	PC1	PC2	PC3	PC4	PC5	PC6
Eigenvalue total	4.262	0.887	0.407	0.343	0.083	0.018
Variability (%)	71.036	14.787	6.783	5.709	1.385	0.301
Cumulative (%)	71.036	85.822	92.605	98.314	99.699	100.000
Variables	Eigenvectors of the components					
BDM (mm)	0.430	-0.161	-0.582	-0.277	0.543	0.281
BT (mm)	0.444	-0.247	-0.225	-0.333	-0.738	-0.187
AT (sqmm)	0.436	-0.220	0.261	0.566	-0.148	0.592
AnTS^−1^	0.235	0.907	-0.252	0.134	-0.172	0.104
TBAS^−1^ (sqmm)	0.396	0.201	0.690	-0.536	0.193	0.039
BLT	0.464	-0.038	0.047	0.433	0.266	-0.723

## Data Availability

The data information will be available on urgent request of the authorized person only.

## Abbreviations

BJRI: Bangladesh Jute Research Institute
JAES: Jute Agricultural Experiment Station
SPSS: Special Package for the Social Sciences
RCBD: Randomized Complete Block Design
PCA: Principal component analysis
LSD: Least significant differences
GDP: Gross Domestic Product.
